RETRACTED

# Solar-Aligned Pictographs at the Paleoindian Site of Painel do Pilão along the Lower Amazon River at Monte Alegre, Brazil

**DOI:** 10.1371/journal.pone.0167692

**Published:** 2016-12-20

**Authors:** Christopher Sean Davis

**Affiliations:** Anthropology Department, Northern Illinois University, Dekalb, Illinois, United States of America; Université de Poitiers, FRANCE

## Abstract

The archaeological sites near Monte Alegre, along Brazil's lower Amazon River, provide new information on the little-known activities and symbolism of South American Paleoindians toward the end of the Ice Age. While paleoindian sites like Monte Verde in Chile, or Guitarrero Cave in Peru, are located near the pacific coast, Monte Alegre lies much further inland, 680 km upriver from the mouth of the Amazon River and the Atlantic Coast. With excavated wood charcoal radiocarbon dated as early as 13,200 calibrated years ago, the hill—as a source of sandstone and quartz lithics—supplied early pioneers with adequate tools needed for colonizing the interior of the continent. Once there, they painted rock art on the landscape, which bears a record of the sun's horizon positions throughout the year. At just 2° south of the equator, Monte Alegre shows no overt seasonal changes beyond fluctuating rainfall amounts, unlike at higher latitudes where temperature, amount of daylight, foliage, and forms of precipitation markedly change. Near the equator, solar and stellar horizon sightings most visibly track the passage of time and seasonal cycles. However, horizons are often hidden behind high forest canopy throughout much of the Amazon Rainforest; but in the Monte Alegre hill ridges looming above the river, paleoindians could hike above the canopy to peer at the horizon, more effectively synchronizing their activities to ecological cycles. This research suggests that Monte Alegre paleoindians delimited the azimuthal range of the sun in a solar year with notational pictographs aligned to horizon sightings at Painel do Pilão, and leaving a painted grid of tally marks that might have served as a rudimentary early calendar. The broad-reaching implication for early Americans is that through the strategic placement of rock art, these ancient artists fostered predictive archaeorecording from which resources could be optimally extracted, ceremonial activities could be consistently scheduled, and gatherings for social and economic exchange could be more efficiently coordinated.

## Introduction

Approximately fifteen kilometers southwest of the city of Monte Alegre, in the Brazilian state of Pará, ancient rock art sites dot the caves and rock faces of three hilly sandstone ridges that are adjacent to the northern bank of the Amazon River [see 1]. Nearly all of the 600+ images are pictographs painted in red to yellow earth tones and unevenly distributed among fourteen different sites. Four of the fourteen sites are open-air vertical rock walls or outcrops while the remaining ten are in small caves or shallow rock shelters. All the outdoor sites contain individual pictographs as well as panels of grouped paintings. Most of the cave and shelter sites have individual pictographs, except for the outer entryway pictographs at Caverna da Pedra Pintada, which are clustered like panels.

RETRACTED

Anna Roosevelt and her team (1996) excavated at Caverna da Pedra Pintada, the largest and closest painted cave to the Amazon River, on a hill called Serra da Paituna. There they unearthed evidence of a Late Pleistocene paleoindian occupation period associated with numerous paint drops and lumps of pigment, artifacts, black soil, and other food remains radiocarbon dated to 11,280 to 10,170 uncalibrated years before present (13,630–11,705 cal yr BP—OxCal 4.2) [2–4].

This research corroborates Roosevelt's work by unearthing further evidence of a paleoindian rock painting tradition at *Painel do Pilão*, a nearby open-air outcrop approximately 400 meters from Caverna da Pedra Pintada. Evidence consists of an excavated ochre manuport and a buried painted stone among lithic flakes and boulders quarried from a sandstone schist wall, and deposited in the lowest stratigraphic levels of a small shelter. The wall from which rocks were removed serves as a platform for an observer to stand atop to view red and yellow painted pictographs, some of which depict probable sun and sky-themed representations due to their solstice alignments, and a grid pattern with filled-in tally marks. The solar alignment of these paintings, and the dated antiquity of contextual artifacts and features from the excavation, suggest a tradition of naked-eye ethnoastronomy and rock art took place here, and the grid may have served as one of the earliest solar "calendars" in the Americas.

## Painel do Pilão Rock Shelter at Monte Alegre

Monte Alegre is a town on the eastern edge of a geologic dome of Paleozoic bedrock, which is interrupted by Tertiary graben-like sediment in horizontal layers of schist, clayey schist, and very fine-grained quartzite, along with dyke intrusions of diorite. The dome partly redirects the Amazon River, which bends north around the dome's eastern edge, and floods into Lago Grande lake just south of the dome during the rainy season. This makes the Monte Alegre dome a rare location in the Lower Amazon Basin because the hill ridges appear like gently sloping rocky plateaus (Fig 1) from the river.

RETRACTED

**Fig 1:** *Serra do Ererê* Hill as seen from the Amazon River in mid Spring. To ancient navigators on the Lower Amazon River, this hill would be a place to replenish silicified sandstone lithic tools. Photo taken by Chris Davis on May 2, 2011.

For a Paleoindian culture, the hills offered a lithic source for making sandstone, quartz, and chalcedony stone tools. Its microclimate zones would also have offered hunting grounds for diverse land and aquatic game, like turtle, brocket deer, and macaws; its seasonal marshes allowed for relative ease of mobility by canoe navigation; the caves offered shelter; and the peaks offered a vantage point above the rainforest canopy to monitor fluctuating river levels and make horizon sightings to coordinate seasonal subsistence strategies. The rock art and archaeological excavations appear to support this scenario of land use.

## Methods

The excavation At *Painel do Pilão* was carried out in late April and May of 2011 with the field permit granted by CNPQ and IPHAN- Belém, PA under the supervision of Dra. Denise Schaan at the institute: Universidade Federal do Pará, Belém, Brazil and Universidade Federal do Oeste do Pará, Santarém, Brazil". The entire width of the shelter floor, covering approximately 1.6 x 1.8 meters, was excavated to bedrock at a depth of ~2.6 meters by the author, who was assisted by two local residents, and a Brazilian archaeology student. Excavation levels were determined by natural levels evaluated from changes in sediment grain-size, sorting, and munsell soil colors. The total number of specimens excavated were 1,688 stored in a permanent repository at the Universidade Federal do Oeste de Pará in Santarém, Brazil.

Photographs and Brunton compass readings of the pictographs were taken in 2007 and 2008, and additional photos and enhanced photogrammetric techniques were taken in 2010 using a handheld GPS unit and a gigapan panoramic robot, which preserves visual and angular ratios as seen from the platform stage. In 2011, before and during the excavation season, twenty prominent pictographs, and 280 points on the outcrop surface were laser distance measured from the platform stage, and cardinal directions as well as inclination (altitude) readings were verified with a Leica disto 8 laser distance measure and a TopCom theodolite station.

Previous compass readings in 2007–2008 had to be corrected to true north, which for Monte Alegre's magnetic declination in 2008, was a correction of + 18°01’±19’ [verified using 5]. All electronic devices (GPS and Theodolite) were set to automatically correct for true north at the time of reading, however, a variance of 0–5° intermittently reoccurred among the different devices. This variance may have been due to human error, inclination of the units, and local electronic or magnetic interference.

RETRACTED

Radiocarbon dating of gymnosperm wood charcoal was performed by accelerated mass spectrometry at the University of Arizona NSF-Arizona AMS Laboratory in late 2012 and early 2013. Sample masses varied between 0.4 to 1.97 mg. Calibration curves were calculated with OxCal version 4.2.3 (IntCal 09) in 2013 and recalibrated (IntCal 13) in 2016.

## Results

The excavtion yielded a predominance of lithics, with no significant organic ecofacts (other than charcoal) beyond the first level. The second excavation level was mostly sterile. Levels 3 to 5 saw increases in lithic flakes, charcoal stains (but few solid pieces) and groundstone nodules; and despite some yellowish-hued lithics, there were no significant traces of pigment. The base of level 5 marked a significant boundary where large boulders began to be uncovered. One boulders from level 7 was too large to be fully removed from the excavation pit, so it was propped on one end and shifted to one side as excavation continued. The frequency of lithic flakes increased as well in the lowest levels, including lithic clusters confined to distinct regions, microlith debitage clusters, and several individual and clustered lithics that had pigment stains and relatively smooth textures, suggetive that some may have been given surface treatments or polished in their time (Fig 2).

**Fig 2:** Two-piece large curved rock with central rectangular hole. Discovered separate from each other in level 7, the left piece is well-polished on the dorsal side, including its part of the hole. The top edge of the left piece is also sharp, suggesting functional reuse after breakage.

Overall, the lithic industry contains few formal tools, instead favoring convenience and expediency with little evidence of retouch. To this degree the lithics share similarity to those recovered by Roosevelt [2] at Caverna da Pedra Pintada. Exceptions were found in the lowest three levels, however, where surface textures displayed some aesthetic qualities. Rare recognizeable tool forms include some unifacial and rare bifacial axes or adzes with trace evidence suggestive of lashing. A few borers and scrapers were also identified, some of which show possible marginal heat-treatments for hardened edges. In form, at least, these share similarity to Roosevelt's bifaces and "limaces" [2]. However, unlike at Caverna da Pedra Pintada, virtually no recognizeable projectile points were recovered, except perhaps among microliths. No bone, shell, or food artifacts were recovered either, and only a single thin layer of ash in level 6 alludes to campfire use in the pit. Due to the lack of significant retouch and finished formal tools—especially projectile points—the concluding impression is that the shelter served as a small quarry, having no signs of long-term or periodic habitation. A substantial amount of lithic fragments are probably due to surface reduction resulting in the flattening of the platform wall during the period of deposition for levels 6–8.

RETRACTED

At *Painel do Pilão*, pictographs are positioned in two orientations on a ~15-meter-high sandstone schist outcrop; a lower panel of pictographs at about 1.5 meters off the platform ground, and an upper panel near the floor of a narrow ledge (just above the first panel, about 2 meters above the platform ground) that angles upward along the rise of the rock to the northwest (Fig 3). Beneath this northwest rise, a natural rock shelter cuts deeper into the outcrop and is partially protected from natural erosion and rapid sedimentary deposition by the overhanging structure. The floor of this shelter reaches the natural ground about 1.4 meters below the level of the platform ground (Fig 4).

**Fig 3:** *Painel do Pilão Painted Outcrop* with its rock art surface in the center-to-left foreground, and a rocky perch at a distance in the top right background of the photo. The sun intersects this "window" in the early afternoon, about two weeks before and after the winter solstice.

**Fig 4:** *Painel do Pilão* Shelter Floor approximately 1.6 x 1.8 meter area excavated by Davis in May 2011. The left (northeast) wall forms the base of a platform stage from which one can view the rock art. This wall was made straight and flat throughout the depth of the excavation unit, leaving evidence of wall flakes and large boulders in only the lowest stratigraphic levels. The right side wall and overhanging rocks show the unmodified, angular smooth surface of the natural rock.

The northeast wall of the excavation unit forms the base of a horizontal platform on which one can view the rock art above. Peculiar gouged marks on this platform wall were buried under ancient soil strata at a depth of 70 centimeters, the top of excavation level 6. The marks consist of at least 7 deep cuts diagonally angled from top left to lower right when facing the wall, with some cuts being deeper than others, and the cross-section of the cuts being somewhat rectangular (Fig 5). Additionally, the entire platform wall seemed to have been made straight and flat, forming a roughly 90° angle to the platform's top surface. The flattening of the wall makes it a mostly 180° planar surface, but closer inspection reveals the surface is covered with somewhat consistent 1–3 cm—chips and indentations, like crumpled paper. This is in contrast to the very rounded and smooth natural boulder surfaces of the two other shelter walls. The inference, therefore, is that the wall of the platform—and initial painting of the panels viewed while standing atop it—may have been created around the same time, coinciding with the radiocarbon dates of the soil covering the peculiar gouges unearthed at excavation level 6. Further support for this hypothesis is evidenced by large boulders uncovered in the excavation unit beginning from level 6 to bedrock at the bottom of level 8, and that radiocarbon dates from these lowest levels fall within a 500 year range of time.

RETRACTED

**Fig 5:** Platform Wall. This wall forms the base of the platform from which one can observe the rock paintings above (Fig 3). The slanted grooves gouged into the middle lower portion of the wall were buried to a depth of 70 cm from the original surface (the top of excavation level 6). The photo was taken by Davis in May 2011.

Level seven of the excavation yielded an artifact bearing more direct context to the painting period—a large circular stone with clearly discernible red and yellow smears on its surface (Fig 6), buried at a depth of ~90 to 102 cm. Correlation D-stretch software enhances its now faded features to show a circular yellow smear in between two yellowish-red arch-shaped smears, and a thick horizontal red band beneath them. Burned wood was found in-situ, next to the top edge of the stone, and was radiocarbon dated to between 10,993±62 years before present (13,014–12,725 cal yr BP—OxCal 4.2).

**Fig 6:** Painted Circular Boulder excavated from level 7 at *Painel do Pilão*. The photo, taken by Davis (May 2011), is enhanced by correlation D-stretch-lab to make the red and yellow half circles and red smears more discernible. These red and yellow colors are not part of the natural rock, but instead were added to the surface before the rock was buried. Red and yellow pigment are the two colors used in the rock art panels above the rock shelter where this was excavated.

Another artifact supporting an ancient painting tradition was unearthed in level eight; a chunk of raw ochre with roughly 3 x 4 x 5 centimeter dimensions was buried at a depth of 96 cm. It is the largest ochre sample found in the excavation unit, and it must have been transported to the site since nowhere in the immediate vicinity can ochre be found naturally. A wood charcoal sample from slightly north of the ochre, and a few centimeters above the stratum (a depth of 85–90 cm), was radiocarbon dated to 11,148 ±71 years before present (13,135–12,810 cal yr BP—OxCal 4.2).

A total of four ^14^C samples from two adjacent excavation levels (Fig 7) were dated and all found to be consistent and contemporary to Roosevelt's paleoindian dates from Caverna da Pedra Pintada, 400 meters north of *Painel do Pilão* (Table 1). A fifth carbon sample taken from bedrock at the base of level 8 was much older, dating over 30,300 years before present.

RETRACTED

**Fig 7:** Platform Wall Profile showing the wall gouges as well as projections of the excavation levels, the radiocarbon ages of charcoal from their stratigraphic locations, and art-associated artifacts. The size and irregularity of boulders in the lower stratigraphic levels belies the depositional sequence of features. However, the resting base of the three artifacts (red ochre manuport, painted boulder, and the oldest fragment of the two-piece polished bore-hole fragments) lie underneath all the relevant charcoal dates.

**Table 1:** Radiocarbon Dates of Excavated Gymnosperm Wood from *Painel do Pilão*.

Sample ID	Excavated Level	Surface Depth	Mass	14C B.P.	d14C S.D.	Calibrated Dates Before Present
20110106–17	6	~87 (85–89.5)	1.60mg	11,212	±69	13,242–12900
20110107–2	7	~90 (89–91)	0.40mg	10,993	±62	13,014–12,725
20110107–13	7	~82 (80–85)	1.43mg	11,088	±64	13,084–12,792
20110107–14	7	~87 (85–90)	1.97mg	11,148	±71	13,135–12810
20110108–5	8	108 cm	0.07mg	>30,300		

Table 1 All calibrated dates determined from OxCal version 4.3 on February 25, 2016 at (https://c14.arch.ox.ac.uk).

## Archaeoastronomy Pictographs at *Painel do Pilão*

The context of the excavation data gives the impression that the northern wall of the excavation unit is part of a platform stage from which an observer can view the rock art from a specific location at *Painel do Pilão*. When doing so, the painting most central to the observer's field of view is a grid image that has individual boxes marked with mostly repetitive (but some varying) tallies (Fig 8). Roosevelt was the first scholar to consider its potential function as a calendar. Although alternative theories not related to astronomy can not be ruled out, this author tested several calendar theories (solar, lunar, planetary, stellar) and revealed one possible, though not exact, pattern emerging with the intersection of the setting sun to a rocky perch in the near distance above and to the right of the painted outcrop (Fig 9).

**Fig 8:** "Calendar" Tally Grid. The grid contains 49 visible contiguous boxes in columns of 5, 6, and 7 rows. An additional fish-net lattice grid continues on the right-hand side. The true color photo shows that the painting is in mostly red ink, although D-stretch image enhancement reveals that yellow pigment traces over red lines, especially in the four columns seen to the left-hand side. The yellow paint, has faded significantly. D-stretch also enhances faded X-shaped tally marks in some of the central columns that currently appear as vertical lines. This suggests that the current image was retouched sometime in antiquity, perhaps to preserve or restore the original grid image. There is no indication that the grid overlays an entirely different image.

RETRACTED

**Fig 9:** Sky Orientation of Painel do Pilão showing the cardinal directions of the largest grid image, matrix of lollipop shapes, and the beginning image at the far western edge of the outcrop. Also depicted is the sun capture window, which was laser measured from the viewing platform at a distance of 45 meters. It visibly "captures" the sun ~18–20 days before and after the winter solstice if an observer stands on the (12-meter long) platform at least 9 meters away from, while facing, the grid image.

The annual movement of the sun relative to the rocky perch allows for the intersection of the setting sun through the center of the perch approximately 18–20 days before and after the winter solstice (which currently occurs on December 21) about the beginning of the rainy period for Monte Alegre. If each box of the painted grid image represents one day of observing the setting of the sun relative to the rocky perch, 49 days after the day of the winter solstice, the sun sets too far to the north of the rocky perch, entirely missing the structure. The grid painting has 49 total boxes and the center boxes have tally marks that are simply vertical lines. Most other tally marks are crisscrosses. The rocky perch and the grid image might, therefore, have been a way for paleoindians to foretell the winter solstice and the passage of a new year, along with the rainy season, stream and river flooding, and all the ecological renewal cycles that come with them. The fewest number of boxes are empty boxes with no tally mark inside. These boxes might have been left empty on overcast days that were too cloudy for visual observation of the sun.

In close proximity on the wall further south (to the left-hand side when viewing the grid) are pictographs in the shape of circles connected by vertical and diagonal lines (Fig 10). Among the Monte Alegre sites, these lollipop-shaped designs only occur at *Painel do Pilão*, and only near the grid, possibly to further represent contextual imagery of the sun or other sky objects in the cardinal direction they face on the eastern horizon. A cluster of connected "lollipop" images (eight form a matrix) align to 66° azimuth. According to StarryNight^™^ software (Pro Plus version 6.3), the sun rises at that cardinal direction on the day of the summer (northern) solstice (which has only changed ~1° on the horizon from 13,000 years ago due to obliquity, but would have occured on September 10, 11,200 B.C due to precession instead of June 21 today).

RETRACTED

**Fig 10:** “Lollipop” Images to the left of the grid image face 66° azimuth. Sixty six degrees is the furthest north that the sun rises on the eastern horizon, which, by definition, occurs on the day of the June 21st (northern/summer) solstice.

Naked-eye sky-watchers could determine solstice positions on the horizon using simple methods because the northern solstice is defined by the furthest northeast (summer for the northern hemisphere) that the sun will rise on the horizon for the entire year, regardless of which year in history and regardless of how far earth's axis is tilted (24° or 23.5°). On that day, the sun also sets the furthest northwest on the horizon in the evenings. Each day afterwards, the sun rises and sets further south until it reaches the southern (winter) solstice position; for Monte Alegre this is at 113.5° azimuth on the horizon (~114°) today. The platform does not wrap around this far southwest (making the area difficult to access) and the walls here have no rock art except for 6 vertical lines grouped together under a honeycomb-like cluster of small circular alcoves assumed to have been naturally formed in the wall (Fig 11). These red-painted lines face approximately 112–114° (difficult to pinpoint due to the terrain).

**Fig 11:** Six long vertical lines were drawn at the far left edge of the southeastern wall, beyond vision from the stage and at difficult accessibility. These lines face ~114°, which is the position that the sun rises on the day of the southern (winter) solstice. Presently, trees and vegetative overgrowth block view of the horizon.

However, it is near this same time of year that the setting sun begins to intersect the rocky perch in the distance as seen from the platform stage (see Figs 3 and 9). If the main grid image represents a tally of these sunset intersections near the southern solstice, and the lollipop images are positioned to track sun rises on the northern solstice, the rock art context implies that the artists tracked the daily movement of the sun across the sky—delineating a solar year (Fig 12).

**Fig 12:** Delineating a solar year through rock art at Painel do Pilão as seen relatively from a bird's eye perspective looking down. Not drawn to scale, the grey rectangle represents the cardinal orientation and position of the excavation and the hypothesized sky-themed rock art and tallies The yellow lines represent the path of the sun on the days of the winter and summer solstice, and the equinoxes.

RETRACTED

A third astronomy alignment occurs with a single red pictograph discovered above the excavation unit on a vertical ledge on the underside of the painted outcrop. The ledge may have been intentionally altered, but further investigation is needed for certainty. The painted circle itself faces 270°, but the shelter walls block all views of the western horizon or sky from this location. However, just beneath the circle and ledge is an opening that allows one to see through to the other side of the outcrop and the horizon beyond (Fig 13). This vantage point beneath the painted circle aligns to ~90°, the position of the rising sun on the equinox, which occurs on March 20 and September 23 currently.

**Fig 13:** Red shelter circle above the excavation unit, but underneath the painted outcrop. The circle faces 270° but the shelter prevents view of the western sky. However, beneath the red circle is a crevice that allows view of the eastern sky. The red circle marks a spot where the sun would shine through the crevice directly beneath the circle on the day of the equinox.

## Discussion

A few rock art sites from the terminal Pleistocene to early Holocene periods have been recently discovered in Brazil [4, 6–9]. Other sites, presumed to be more recent, have been investigated for their potential archaeoastronomy alignments as well [10], like the megaliths near Calçoene, Amapa [11], or the prolific grooves and cupules at Pedra da Inga in Paraiba [12].

Yet, the most interesting similarities to Painel do Pilão rock art can be found among the São Francisco art tradition from site: BA-RC-28, located in Coribe, Bahia—Brazil. There, pictographs depict numerous long vertical lines and rectangular grids that similarly may reflect a tally system of sky observations [13–15]. Even as far south as Santa Catarina Island in Florianopolis, Brazil, some rock art petroglyphs may depict tallies and diamond lattice patterns—theorized [16] to represent fishing nets—do share compositional similarities to the right-side portion of the Painel do Pilão grid.

Another stylistic and motif-themed similarity is found among the Agreste tradition from Pedra do Velho, Samuel in Paraiba, Brazil, where 3-digit stick figures of probable turtles and lizards are depicted crowding around a concentric circle [13, 14]. These drawings are similar to some of the zoomorphic pictographs at Painel do Pilão and throughout Monte Alegre rock art sites, especially at the other open-air site named Mirante.

A number of other pictograph motifs throughout Monte Alegre share some similarities to rock art sites throughout Pará, Brazil [17] but many of those similarites can be seen in the posture of the humanoid stick figures. There seem to be less sky-themed images at other Pará sites, and several sites have petroglyphs instead of pictographs. Regardless, although specific dates remain elusive, the dispersal of sites suggest a widespread practice of shared knowledge and artistic influences [6, 17].

RETRACTED

In no way can or should all the images at Painel do Pilão be considered to have preserved since the paleoindian period 13,000 years ago. Image enhancements of the grid shows evidence of earlier designs, but currently there is no way to determine how much time elapsed between overlapping paint strokes. The excavation recovered lithic deposits in nearly all levels but the few reliable charcoal samples from higher levels have not yet been analyzed. Charcoal from wall fall, that almost certainly fell from close to the surface, was dated to 2,112 ± 40 yr BP (2251–1989 cal yr BP OxCal 4.2 IntCal09). Therefore it is likely that some painted images (possibly the 12 yellow handprints overlaying the red pictographs on the lower panel) were produced recently. However, the data presented here lays a case for initial painting to have begun around the time that the area was first inhabited 13,000 years ago, and that those earliest images, which were probably retouched or traced more recently, were position in the most prominent wall locations and height visible from the stage. These images have, and are somewhat bound by, the horizon azimuthal markings of sunrises and possibly sunsets between solstices in a solar year.

While a matrix of lollipop images, and a few others that are paired, align to 66° azimuth, a few single isolated lollipop images (5 out of 18 total) do not, therefore, the motif might not represent the sun. They could represent certain stars along the ecliptic, planets, the moon, or constellations; all these theories (especially Mercury and Venus) the author explored with the StarryNight sky simulator but found little correlation.

Another alternative theory difficult to test is that the lollipop images represent the maracas of individuals who may have pilgrimaged to the site. Maracas are sited as being symbolically and spiritually vital to contact period Brazilian cultures [18, 19], utilized by shaman [20], but also by layman during dances and ceremonies [21, 22]. However, if they represent maracas—symbolic of personal identities—we might expect them to be adjacent to similar personal identifiers, like the twenty-in-all red and yellow painted handprints; yet, they are not. Also, this alternative theory does not address why 13 of the 18 lollipops align near the solstice sunrise. Of the other 5 lollipops, two on the upper ledge face the sun as it rises higher in the sky during the days around the same solstice, and a third one, located north of the grid on the lower panel, is not a "true" lollipop" because it is "animated" by the addition of horns and legs. Therefore, the horizon sun assignments provide the strongest evidence, further strengthened by the painted red equinox circle.

RETRACTED

The painted circle underneath the outcrop above the excavation unit is oriented to ~90°, and under initial considerations it is difficult to understand how the equinox would have been determined by naked-eye astronomers unless they had counted the total number of days between solstices to compute the half-way mark.

Ethnographic accounts of Amazonian indians suggest that more importance was given to the day of the year when the sun cast no shadow from a gnomon at midday [23, 24]. Such an event only occurs for just one day of the year near midday when the sun passes through the exact zenith of the sky for a given location that must lie near the equator at lattitudes between the tropics. Monte Alegre, at 2°3' south, meets this criterion. However, the day this occurs there is not on the day of the equinox. Presently, this day of virtually no shadow occurs on March 15 and September 28, about seven days away from the equinox. On these days at about 12:28 PM, the sun reaches the exact zenith at 89.9° altitude [calculated for the year AD 2010 from the 25], casting virtually no shadows. On those days, however, the sun rises on the horizon at ~92°, not 90°. Even 13,000 years ago, according to StarryNight software's reconstructed ancient sky, the sun would have rose in the morning at 91.48° local azimuth on the day it passed exactly through the zenith, thereby casting no shadows (accounting for obliquity and precession). Neither ancient nor modern dates for the shadow phenomenon occur on the equinox, and neither coincide with a horizon alignment of 90°. That alignment occurs on the day of the true equinox, so the painted circle must truly have been placed to mark sunrise on the day of the true equinox, however and whenever the artists painted it there.

## Conclusion

Recognizing the passage of the seasons is perhaps something taken for granted in the northern or far southern latitudes because there are so many obvious signs. However, tropical environments—like at Monte Alegre just 2° south of the equator—do not have any of those telltale higher lattitude signs. There are no major changes in temperature, no changes of precipitation from rain to snow, no significantly shorter or longer days and nights, and no widespread coordinated shedding or color change of tree foliage. Therefore, the passage of the seasons—i.e. a solar year—is perhaps most recognizable by tracking the migration of the sun between southern and northern solstices. To do this, however, one needs a clear view of the horizon—which is usually difficult in a rainforest environment—but Monte Alegre provides the necessary elevation above the forest canopy to view the horizons.

RETRACTED

For paleoindian cultures, the river would have been the most efficient mode of travel, the hills at Monte Alegre offered lithic tools and horizon sightings, and once there, tracking the sun through rock art pictographs and tally marks allowed for them to mark the cyclic passage of time in a rudimentary calendar. Armed with this visual aide, the ancient Amazonians could better predict and schedule subsistence and social activities, like resource acquisition and ritual ceremonies.

The results of this research have implications on the development of traditional astronomy knowledge systems extending to the terminal Pleistocene. This was a critical moment in history when our human ancestors were faced with rapid changes to the global climate. We do not know the extent to which paleoindians recognized these changes, but it is during this time period that Monte Alegre first shows evidence for paleoindians using rock paintings. I've argued here that the context of the rock paintings indicate a method of recording seasonal sky observations in pictographs with enough precision that it could have helped them predict cyclic patterns of resource availability in the local environment.

Archaeoastronomy sites like at Painel do Pilão are pushing further back in antiquity the evidence for human use of astronomy observations to marke the passage of time. And even though specific rock drawings can not be pinpointed to over 13,000 years ago, this research helps establish that tropical cultures engaged and utilized sophisticated knowledge of astronomy maintained through rock art and possibly shared or reimagined by more recent cultures who either inherited or rediscovered the ancient paintings as they traveled far afield throughout eastern South America.

Beyond the art and archaeoasronomy, the recovery of lithics and the reduction of a platform wall during the paleoindian period shows that the interior of the South American continent was being inhabited as early or earlier than many coastal sites. And the preence of rock art during that initial period suggests that rock art as a form of archaeorecording may have been an adaptive strategy consistent with pioneers who sought to familiarize themselves to a new landscape.

Similar astronomy lore [26–28] is found among more recent cultures for village orientation and construction in Amazonia [24, 29–32] and the Andean regions of South America [33–36], for the layout of many platform plaza constructions in Mesoamerica [26, 37–39], and for the medicine wheels, gnomons, and sun dagger rock art of Sun-watcher chiefs in North America's southwest and plains cultures [40–43].

RETRACTED

## Supporting Information

S1 File Supporting Data Ser. A compilation of individual data sets, including excavation catalog, AMS carbon sample reports, and Sun alignment data tables.
(PDF)

## References

[1] PereiraE. A Arte Rupestre de Monte Alegre, Pará, Amazônia, Brasil. Belém: Museu Paraense Emílio Goeldi; 2012.

[2] RooseveltAC, Lima da CostaM, MachadoCL, MichabM, MercierN, ValladasH, et al Paleoindian Cave Dwellers in the Amazon: The Peopling of the Americas. Science. 1996;272(5260):373–84.

[3] RooseveltAC. The Development of Prehistoric Complex Societies: Amazonia, A Tropical Forest. Archeological Papers of the American Anthropological Association. 1999;9(1):13–33.

[4] RooseveltAC, DouglasJ, BrownL. The Migrations and Adaptations of the First Americans: Clovis and PreClovis Viewed from South America In: JablonskiNG, editor. The First Americans: The Pleistocene Colonization of the New World. 27 Berkeley: Memoirs of the California Academy of Sciences; 2002 p. 159–236.

[5] NCEI NCfEI. Magnetic Field Calculators Boulder, Colorado: National Oceanic and Atmospheric Administration (NOAA) Satellite and Information Service (NESDIS); 2016 [updated September 1 2016 14:29:26 UTC; cited 2016 October 15].

[6] NevesWA, AraujoAGM, BernardoDV, KipnisR, FeathersJK. Rock Art at the Pleistocene/Holocene Boundary in Eastern South America. PLoS ONE. 2012;7(2):e32228 doi: 10.1371/journal.pone.0032228 2238418710.1371/journal.pone.0032228PMC3284556

[7] JorgeM, ProusA, RibeiroL. Brasil Rupestre: Arte Pre-historica brasileira. Curitiba, Brazil: Zencrane Livros; 2007.

[8] GuidonN. Arqueologia da região do Parque Nacional Serra da Capivara—Sudeste do Piauí. São Raimundo Nonato, PI 2003.

[9] ProusA, FogaçaE. Archaeology of the Pleistocene-Holocene boundary in Brazil. Quaternary International. 1999;53:21–41.

[10] BeltrãoMCDJN, R. MesquitaS. S., BomfinM. T. M. P. Les représentations pictographiques de la Serra da Pedra Calcaria: Les Tocas de Buzios et de Esperança. L’Anthropologie 1990;94(1):139–54.

[11] CabralMP, de Moura SaldanhaJD. Paisagens megalíticas na costa norte do Amapá. Revista de Arqueologia. 2009;21(1).

[12] PavíaAF. La Itacoatiara de Ingá, un registro astronómico. Agrupación Astronómica de la Safor. 2005;53.

[13] Martin G. Pré-história do Nordeste do Brasil: Editora Universitária UFPE; 1997.

[14] EtchevarneC. A ocupaçao humana do Nordeste brasileiro antes da colonizaçao portuguesa. Revista Usp. 2000; (44):112–41.

RETRACTED

[15] ProusA. Arqueologia Brasileira. Brasília: Universidade de Brasília; 1992.

[16] AguiarR. A arte dos pescadores pré-historicos no litoral catarinense. Ensaios interpretativos sobre a arte rupestre na Ilha de Santa Catarina e ilhas adjacentes. Revista Multitemática das Faculdades Energia. 2004:91–100.

[17] PereiraE. Arte Rupestre Na Amazonia Para. UNESP, editor. Belem: Museu Paraense Emilio Goeldi; 2002.

[18] SoutheyR. History of Brazil: Part the First. London: Longman, Hurst, Rees, and Deme, Paternoster row; 1810.

[19] JdLéry. History of a Voyage to the Land of Brazil, Otherwise Called America. Berkeley, CA: University of California Press; 1992.

[20] RothWE. An Inquiry into the Animism and Folk-Lore of the Guiana Indians. Washington D.C: Buereau of American Ethnology; 1915 103–386 p.

[21] WallaceAR. A Narrative of Travels: Amazon and Rio Negro, with an account of the native tribes. 2nd edition ed London: Ward, Lock and Co; 1889.

[22] WhiffenT. The North-west Amazons: Notes of Some Months Spent Among Cannibal Tribes. London: Constable and Company, Ltd; 1915.

[23] FabianSM. Patterns in the Sky: An Introduction to Ethnoastronomy. Prospect Heights, Illinois: Waveland Press, Inc; 2001.

[24] Reichel-DolmatoffG. Astronomical Models of Social Behavior Among Some Indians of Colombia In: AveniAF, UrtonG, editors. Archaeoastronomy in the New World: American Primitive Astronomy. United Kingdom: Cambridge University Press 1982 p. 165–81.

[25] Astronomical Applications Department. Sun or Moon Altitude/Azimuth Table Washington, DC 20392–5420: U.S. Naval Observatory [updated 24 July 2015 13:0; cited 2016 October 15]. Form B—Locations Worldwide: [http://aa.usno.navy.mil/data/docs/AltAz.php.

[26] AveniAF. Empires of Time: calendars, clocks, and cultures. New York: Basic Books; 1989.

[27] AveniAF. Circling the Square: how the conquest altered the shape of time in Mesoamerica. Philadelphia, PA: American Philosophical Society; 2012.

[28] ZuidemaRT. Anthropology and Archaeoastronomy In: WilliamsonRA, editor. Archaeoastronomy in the Americas. College Park, MD: Ballena Press Center for Archaeoastronomy; 1981 p. 29–31.

[29] FabianSM. Space-Time of the Bororo of Brazil. Gainesville: University Presses of Florida; 1992.

[30] UrtonG. At the Crossroads of Earth and Sky: An Andean Cosmology. Austin: University of Texas Press; 1981.

[31] Wilbert J. Warao Cosmology and Yekuana Roundhouse Symbolism. In: Magaña E, Mason P, editors. Myth and the Imaginary in the New World. CEDLA Latin American Studies. Amsterdam: CEDLA Latin American Studies; 1986. p. 427–58.

[32] MagañaE, MasonP, editors. Myth and the Imaginary in the New World. Amsterdam: CEDLA; 1986.

RETRACTED

[33] KelleyD, MiloneE. Exploring Ancient Skies: A Survey of Ancient and Cultural Astronomy. 2 ed New York: Springer; 2011.

[34] TruelLR. Canto Grande y su Relación con los Centros Ceremoniales de Planta en “U” Arqueología de la Costa Central. Talleres de Mundo Gráfico SA, Ind. Lima, Peru: Santa Rosa; 1997.

[35] AveniAF. The Lines of Nazca. Philadelphia, PA: American Philosophical Society; 1990.

[36] MalatestaP. The Nazca Mystery. UNESCO Courier. 1998;51(3):44–9.

[37] Evans ST. Ancient Mexico and Central America: archaeology and culture history: Thames & hudson; 2013.

[38] AveniAF. Skywatchers of Ancient Mexico. Austin: University of Texas Press; 1980 356 p.

[39] TedlockB. Maya Astronomy: what we know and how we know it. Archaeoastronomy. 1999;14(1):39–58.

[40] SofaerA, SinclairRM. Astronomical Markings at Three Sites on Fajada Butte In: CarlsonJB, JudgeWJ, editors. Astronomy and Ceremony in the Prehistoric Southwest. Maxwell Museum of Anthropology Anthropological Papers. Albuquerque, NM: University of New Mexico; 1983.

[41] KruppEC. Archaeoastronomy unplugged: eliminating the fuzz tone from rock art astronomy In: HamannD, editor. International Rock Art Congress 1994. American Indian Rock Art 3. 21 ed Phoenix: American Rock Art Research Association; 2006 p. 353–70.

[42] BraceGI. Boulder monuments of Saskatchewan. Saskatoon: Saskatchewan Archaeological Society; 2005.

[43] TitievM. Old Oraibi, a study of the Hopi Indians of third mesa. Cambridge, Mass: Harvard University Museum; 1944 xi, 277 p. p.

